# Construction Means of Soil Microbial Synusiologic Network Based on ANN

**DOI:** 10.1155/2022/1708350

**Published:** 2022-10-03

**Authors:** Xia Li, Huixian Wang, Miaoxin Yuan

**Affiliations:** ^1^College of Mechanical and Vehicle Engineering, Taiyuan University of Technology, Taiyuan, Shanxi 030024, China; ^2^Shanxi Academy of Agricultural Science, Shanxi Agricultural University, Taiyuan, Shanxi 030031, China; ^3^China Energy Conservation DADI (Hangzhou) Environment Remediation Co Ltd, Hangzhou, Zhejiang 310020, China

## Abstract

With the construction of synusiologic civilization and synusiologic environmental protection entering a new era driven by data, the breadth and depth of application of the DM technique in the domain of synusiologic environmental protection are constantly strengthened. If reasonable planning is not carried out in the process of social construction, it will cause unpredictable damage to the synusiologic environment. However, traditional synusiologic planning means too much human interference, and there are still some shortcomings in accuracy and operability, which means they cannot guide synusiologic construction well. In order to analyze the contribution of the soil nutrient data to soil fertility and dig out the knowledge describing soil fertility, this paper studies the construction means of soil microbial synusiologic network by ANN. By simulating the learning, memorizing, and processing problems of human brain neurons, the artificial network establishes a parallel distributed processing system computing DMG model with a large number of connections, which can quickly acquire knowledge from the outside world and store and process it and respond to the changes in the external environment in time. According to the research in this paper, the network performance of this algorithm is 18% better than that of the traditional algorithm, and it is suitable to be widely put into practice.

## 1. Introduction

With the rapid improvement of social eco, the intensity of land use in China is increasing year by year, and the soil pollution caused by it is becoming more and more prominent and serious [1]. Land is the source of the basic means of subsistence for human beings. The advancement of message technique, in the complex production system in agricultural production makes the soil fertility level highly uncertain, which has a great impact on the growth of crops [2]. The DM technique is a process of classifying and extracting massive data, discovering the interrelations among them, and generating new rules [3]. The purpose of the DM technique is to analyze the relationship between data from multiple dimensions, search for the message hidden in the data, provide decision support for scientific research, and promote the transformation of production and lifestyle. In order to understand the overall situation of soil pollution and remediation, study the mutual influence of various factors in the domain of soil remediation [4]. At the same time, synusiologic civilization construction and synusiologic environmental protection have entered a new era driven by data [5]. The data collected in the work of resolutely fighting the battle against pollution, continuously improving the quality of the synusiologic environment, and constantly meeting the people's growing beautiful synusiologic environment are often incomplete, unclear, large, and random, so they cannot be separated from the support of the DM technique [6]. The concept of a synusiologic network in ecology has a long history and was put forward in 1859. Nowadays, synusiologic network, as a branch of ecology, mainly studies the complex structure and interaction among species, explores the temporal and spatial variation laws, clarifies the internal structure of complex systems, analyzes the specificity of different ecosystems, and then discusses the ways and strategies to keep the sustainability of natural systems [7]. At present, the city is in a period of rapid improvement and construction. However, in the process of urban improvement and construction, the problem of urban construction's consumption and destruction of synusiologic background has become more and more serious, and the fragmentation of a large number of agricultural and forestry green spaces has greatly affected the urban natural synusiologic landscape [8]. Since the 1990s, the concept of synusiologic network has been studied and applied by many disciplines, such as ecology, geography, and planning, and the knowledge of synusiologic network in various disciplines has been continuously integrated, which has enriched the connotation of synusiologic network and made the expression of form and structure more and more clearly visible [9]. In the process of urban improvement and people's daily life, the existence of green space has important value and significance. It can optimize the spatial pattern of cities, support the improvement and construction of cities, improve the synusiologic environment of cities, provide a good living environment for human beings, etc., so it is very important for the planning and construction of urban green space [10]. The technical level has always restricted the improvement of land use, and the industrial revolution has promoted the application of nature protection and synusiologic network thought in the planning domain [11]. From the end of the 19th century to the beginning of the 20th century, natural landscapes began to become the content of urban planning. The second industrial revolution transformed cities and villages, and seminatural areas began to be transformed into agricultural land and expanded continuously. Since the end of the 20th century, the establishment of national parks and nature reserves has become the main way to slow down the extinction of species and the decline of natural ecosystems [12]. In the process of urbanization, the construction of a synusiologic civilization cannot be ignored. The function of the synusiologic environment plays a vital role in the improvement of urban and rural areas, including protecting biodiversity, reducing pollution and noise generated in the process of urban improvement, reducing the urban heat island effect, and other functions.

The innovation of this paper lies in the following:

1. The ANN is introduced. This is the algorithm of this paper, so it is necessary to discuss it. ANN is a computing model of a parallel distributed processing system, which is established by simulating the learning, memory, and problem solving functions of human brain neurons. It can quickly acquire knowledge from the outside world and store and process it and respond to the changes in the external environment in time.
2. The application of ANN to a synusiologic network is introduced. This is a discussion around the theme of this article. It is feasible to apply synusiologic ANN to the evaluation or identification of synusiologic environmental quality. At the same time, because of its excellent properties, such as self-organization, self-adaptation, self-learning, and fault tolerance, and its complex parallel distributed processing ability, it can accurately evaluate the synusiologic environment quality from the specific learning samples.
3. The model construction is discussed. Let readers have a certain understanding of this principle. Ecological environmental quality evaluation is essentially a pattern recognition problem, that is, the actual monitoring results of the synusiologic environmental quality evaluation index system are compared with the array of corresponding synusiologic environmental quality evaluation standard values, and the synusiologic environmental quality grade corresponding to the standard value array closest to the array of monitoring values is the recognition result of the BP ANN model, that is, the synusiologic environmental quality evaluation result of the corresponding area.

This paper is divided into five parts: The first part is the background and brief introduction of this paper; the second part is related research and the introduction of this paper. The third part is at the means adopted and the discussion of this research. The fourth part, which is the core of this paper, is the construction of relevant theories and models. The fifth part is the conclusion.

## 2. Related Work

Li established a two-level BP network model for urban comprehensive environmental quality evaluation, in which the first-level evaluation established BP network models for three subsystems atmosphere, surface water, and noise and evaluated the atmospheric environmental quality, surface water environmental quality, and acoustic environmental quality [13]. Wu suggested that qualitative research be adopted. By studying the public perception of the Chicago River synusiologic corridor, it was found that six elements of the green space synusiologic network, nature, art, cleanliness, safety, improvement power, and proximity, have a direct influence on the public perception of the green space synusiologic network [14]. Schütz suggested that landscape ecology is a new branch that extends from ecology, taking the landscape as the object and applying synusiologic principles to study the spatial structure, function, and dynamic changes of the landscape in a large enough area [15]. Taghizadeh-Mehrjardi suggested quantitative research and found that the vegetation types and the degree of protection on both sides of the river bank have a great influence on public perception [16]. Xie suggested that the BP network should be used for comprehensive evaluation of urban environmental quality, and the nonlinear relationship between the urban environment and its influencing factors was established to evaluate the grade of urban environmental quality [17]. Mandakovic suggested that 433 typical cases of greenbelt synusiologic networks in Northern Ireland, Scotland, England, and Wales should be investigated by a questionnaire, which aimed at the definition, current situation, and a local greenbelt synusiologic network project, etc., so as to determine the public's understanding of greenbelt synusiologic networks [18]. Yu suggested that the atmospheric environmental quality evaluation model based on the BP network should be established, and the model should be used for atmospheric environmental quality evaluation, and the evaluation results were compared with those of fuzzy mathematics evaluation means, which showed that BP ANN was universal, reasonable, and practical [19]. She suggested that, based on regional land cover, synusiologic evaluation, wildlife protection, and other objectives, corridors and networks should be regarded as the framework of the green space synusiologic network for overall planning, and important patches should be selected as synusiologic nodes through node weight analysis, and seven different network schemes should be formed after synusiologic corridors are connected, then the network structure index of each scheme should be calculated, and finally the best scheme can be obtained by analyzing and comparing them [20]. Li suggested using the BP network model to evaluate the atmospheric environmental quality of a city and compared the evaluation results of this means with fuzzy decision, grey clustering, and comprehensive evaluation means, which proved the superiority of the BP network model in atmospheric environmental quality evaluation [21]. Zhang suggested that the landscape structure index should be applied to the evaluation of urban green space synusiologic network, and the corridor index, patch index, and matrix index should be used to optimize it through comprehensive analysis [22]. It is suggested that the BP network should be applied to lake water quality classification, and the water quality index data of 25 lakes in China should be used as training samples. Zhang established a water quality classification model and used the model to classify the water quality of 6 lakes [23, 24].

The rapid improvement of China's cities has led to the continuous expansion of construction land, which has led to the increasingly broken landscape blocks of urban green space, which has a negative impact on the synusiologic function of the whole city. The synusiologic function of urban green space is closely related to the urban landscape, and the construction of landscape pattern is crucial to urban synusiologic construction. It is very important to establish an ecosystem simulation and prediction model, but it is often difficult. It is of great significance to study the construction means of soil microbial synusiologic network based on ANN in this paper.

## 3. ANN

### 3.1. Overview of ANN

With the improvement of science and technique, computers have been widely used for their powerful computing power and message processing power. However, in terms of perception, pattern recognition, and decision-making problems, the processing ability of computers is not as good as that of people. DM is the process of extracting hidden, unknown but potentially useful messages and knowledge from a large number of incomplete, noisy, fuzzy and random practical application databases. In today's message age, people are eager for ever-changing messages. At present, in the transaction records and financial statements in various enterprises and commercial domains and the data collected in scientific research domains (for example, meteorological images returned by meteorological satellites), the data scale is often tens of megabytes, or even hundreds of gigabytes. The DM technique based on the neural network is to explicitly express the knowledge implied in the neural network in an easy-to-understand way. People began to study the organizational structure and operation mechanism of the human brain, hoping to find a new means of message display, storage, and processing by imitating the human brain and design a brand-new processing structure model, which prompted the birth of the artificial neural network (ANN) research algorithm. The structure of the BP neural network is shown in Figure 1.

The BP neural network result algorithm is as follows:

The network has *I* nodes in the input layer, *J* nodes in the hidden layer, and *K* nodes in the output layer. Let *x*_*p*_=(*x*_*p*1_, *x*_*p*2_,…, *x*_*pI*_) represent the network input, and *O*_*p*_=(*o*_*p*1_, *o*_*p*2_,…, *o*_pk_)′ and *T*_*p*_=(*t*_*p*1_,…, *t*_pk_)′ represent the actual output and expected output of the network, respectively, where *p*=1,2,…, *P* and the number of samples is *P*. (*o*_*p*1_′, *o*_*p*2_′,…, *o*_*pJ*_′) denotes the output of hidden layer nodes, *w*_ij_′ denotes the weights of the *i*(*i*=1,2,…, *I*)th input layer node to the *j*(*j*=1,2,…, *J*)th hidden layer node, and *w*_jk_ denotes the weights of the*j*th hidden layer node to the *k*(*k*=1,2,…, *K*)th output layer node.

The excitation function of the network is *f*(*x*)=1/1+*e*^−*x*^, then for the *p*nd sample, there are the following:

The output of the hidden layer of the network is

(1) $$\begin{array}{c} o_{pj}^{\prime }=f\left(net_{pj}\right)=f\left(\overset{l}{\underset{i=1}{\sum }}w_{ij}^{\prime }x_{pi}\right),j=1,2,\ldots ,J. \end{array}$$

The output of the output layer of the network is

(2) $$\begin{array}{c} o_{pk}=f\left(net_{pk}\right)=f\left(\overset{J}{\underset{j=1}{\sum }}w_{jk}o_{pj}^{\prime }\right),k=1,2,\ldots ,K. \end{array}$$

So far, BP network has completed the approximate mapping of *I*-dimensional space vector to *K*-dimensional space.

Using the square error function, the error of the *p*th sample is

(3) $$\begin{array}{c} E_{p}=\frac{1}{2}\overset{K}{\underset{k=1}{\sum }}{\left(t_{pk}-o_{pk}\right)}^{2},p=1,2.\ldots ,P. \end{array}$$

For*P* samples, the global error is

(4) $$\begin{array}{c} E=\frac{1}{2}\overset{P}{\underset{p=1}{\sum }}\overset{K}{\underset{k=1}{\sum }}{\left(t_{pk}-o_{pk}\right)}^{2}=\overset{P}{\underset{p=1}{\sum }}E_{p}. \end{array}$$

Synonyms similar to DM include data fusion, data analysis, and decision support. From this definition, we can realize that the following data must be true, abundant, and noisy discoveries, which are knowledge discoveries that users are interested in. Knowledge should be acceptable, understandable, and applicable, which does not require the discovery of universal knowledge but only supports specific discovery problems. Modern computer and database techniques can already support the storage and quick retrieval of such a database. This means that we have the ability to transform such “data floods” into “orderly” but “mountain-like” data sets. The DM technique of neural network integrates parallel intuition and serial logic and seeks an unknown message by learning the known message. It is suitable for nonlinear data and noisy data, especially when fuzzy, imprecise, and incomplete knowledge (data) is the feature, or there is no clear mathematical algorithm to analyze the data, it can achieve the effect that traditional symbolic learning means cannot achieve. ANN is a computing model of a parallel distributed processing system, which is established by simulating the learning, memory, and problem-solving functions of human brain neurons. It can quickly acquire knowledge from the outside world, store and process it, and respond to the changes in the external environment in time.

In a broad sense, data and messages are also forms of knowledge, but people regard concepts, rules, patterns, rules, and constraints as knowledge and data as the source of knowledge. Original data can be structured data such as relational databases, semi-structured data such as text, images, or even heterogeneous data distributed on the network. However, in the face of “mountain-like” data collection, the traditional data analysis means are difficult to cope with in terms of time and space, and people cannot understand and effectively use such data. With the continuous improvement of various computer management message systems and message technologies, more and more data is being collected into databases at an unprecedented speed. However, due to the huge and complex amount of data and the lack of effective data analysis tools, only a small amount of data will be used, and more will become “data garbage”. With the improvement of ANN research, people's theoretical research on neural networks mainly focuses on using the research results of neural basic theory to explore neural network models with more perfect functions and superior performance by mathematical means.

Many people regard DM as knowledge discovery in a database. The means of knowledge discovery can be mathematical, nonmathematical, deductive, or inductive. The discovered knowledge can be used for message management, query optimization, decision-making knowledge, and process control, etc., and can also be used for the maintenance of data itself. For the current general database management system, all it can do is to make some simple queries and report statistics, which cannot keep up with the needs of the times. Faced with such a huge database, people are more eager to process and analyze these data at a higher level in order to get the general characteristics of the data and forecast the improvement trend. An ANN is a nonlinear dynamic system composed of a large number of parallel distributed processing units. It is very suitable for dealing with nonlinear and noisy data, especially those problems which are characterized by fuzzy, incomplete, and imprecise knowledge or data. These are the problems that DM tools have to face and try to solve.

### 3.2. ANN for Synusiologic Network

The ecosystem is a very complex big system. Whether it is a global ecosystem or a small regional ecosystem such as a watershed or a small reservoir (lake), its complexity is not only manifested in the structure of the ecosystem but also in the influencing factors of the ecosystem. Therefore, it is generally difficult to establish a more accurate mathematical model. However, due to the need for research, sometimes we have to overcome this difficulty and try to establish a reliable and easy-to-use quantitative model. The ecological environmental quality evaluation is one of the important means of synusiologic environmental management. Through environmental quality evaluation, the synusiologic environmental quality of a certain area can be scientifically evaluated, and a scientific basis can be provided for synusiologic environmental management, synusiologic environmental engineering, formulation of synusiologic environmental standards, synusiologic environmental planning, and synusiologic environmental construction.

A comprehensive evaluation of synusiologic environmental quality is based on the regional synusiologic environmental investigation, aiming at the characteristics of the eco-environment in this region, selecting certain evaluation indexes to evaluate by mathematical means, so as to identify the synusiologic environmental quality status and existing problems of different evaluation units and put forward countermeasures for comprehensive treatment. The ecological environmental quality evaluation is an identification process of comprehensively comparing the monitoring data of each index of the evaluated object with all levels of standards to see which level is closest to it. Many people have studied the identification and evaluation of synusiologic environmental quality. It is feasible to apply synusiologic ANN to the evaluation or identification of synusiologic environmental quality. At the same time, because of its excellent properties, such as self-organization, self-adaptation, self-learning, and fault tolerance, and its complex parallel distributed processing ability, it can accurately evaluate the synusiologic environment quality from the specific learning samples.

The traditional synusiologic environment monitoring means are to set up a monitoring system covering the whole area, which mainly uses artificial ground observation, measurement, positioning monitoring, and laboratory analysis to obtain various statistical indicators and comprehensively evaluates the regional synusiologic environment. With the improvement of satellite remote sensing and the characteristics that remote sensing images can quickly provide synusiologic environment messages, the synusiologic environment remote sensing monitoring means have been widely used, from a single factor investigation and monitoring of a synusiologic environment to a comprehensive evaluation supported by multiple data. ANN is widely connected by a large number of simple neurons. It relies on computers to acquire superb computing power, and through the complex network system that simulates the thinking mode of the human brain, it makes use of accumulated knowledge to acquire recognition and association abilities similar to those of human beings.

Because of the complexity of the relationship between input and output in the ecosystem, it is generally reluctant to establish a simple mathematical model. The nonlinear relationship between synusiologic environmental quality and synusiologic environmental index requires the synusiologic environmental quality extraction model to have the function of nonlinear function fitting. The ANN means can handle the nonlinear relationship among variables well, solve the above problems in synusiologic environment quality message extraction, and provide a new technical means for regional synusiologic environment classification message extraction based on remote sensing. The ANN means have made some progress in regional synusiologic environment classification and are an important application of neural network pattern recognition. ANN has been widely used in the domains of system identification and pattern recognition and has made some progress. The ecological environmental quality evaluation is essentially a pattern recognition process, so it is feasible to apply ANN to a synusiologic environmental quality evaluation or recognition. At the same time, because it has excellent properties such as self-organization, self-adaptation, self-learning, and fault tolerance, as well as complex parallel distributed processing ability, it can obtain the weights based on objective data from specific learning samples, and evaluate the synusiologic environment quality more accurately.

## 4. Soil Microbial Synusiologic Network and Its Construction

### 4.1. Soil Microbial Synusiologic Network

A soil ecosystem is a whole composed of the interaction between organisms and the nonchemical environment in the soil through energy conversion and material circulation. The soil ecosystem includes soil minerals, soil organic matter, soil organisms, soil water, and soil air, among which soil microorganisms are the main components of the soil ecosystem. Traditional analysis of microbial community diversity and structure in soil ecosystems is mostly to isolate and culture microorganisms, and then analyze them through general biochemical traits or specific phenotypes, which are limited to isolating microorganisms from the solid culture medium. With the research on the in-situ living state of microorganisms in the soil, it is increasingly found that it is difficult to comprehensively evaluate the diversity of microbial communities by conventional isolation and culture means.

As an important part of the ecosystem, soil microbes play an important role in energy flow, material circulation, soil formation, and maturation, and are one of the sensitive indicators to reflect the changes in the soil ecosystem. Their quantity, population, and composition are important parameters to evaluate soil environmental quality. Soil microorganisms include prokaryotic microorganisms and eukaryotic microorganisms, among which prokaryotic micro-organisms include archaea, bacteria, actinomycetes, cyanobacteria, and myxobacteria, while eukaryotic microorganisms include fungi, algae, and lichens. These microorganisms are the main promoters of nutrient cycling in soil and play a very important role in the soil ecosystem.

Microorganisms in the soil rarely exist alone, but always have more populations gather together. They are mutual environments, influence each other, depend on each other, and repel each other. The knowledge of these interaction laws is soil microbial morphology. Microbial diversity refers to the changes in living organisms at the genetic, species, and ecosystem levels. It represents the stability of the microbial community and also reflects the influence of soil synusiologic mechanism and soil stress on the community. The study of soil microorganisms plays a positive role in understanding the functions of various biological systems. With the improvement of the subject, the research means of microbiology are constantly improved and improved, and new means are constantly emerging.

### 4.2. Construction of Soil Microbial Synusiologic Network

Since the 1920s, the synusiologic function of green space has been paid attention to, which has gradually changed the research of green space from extensive to detailed, from qualitative description to quantitative research. Landscape ecology enables people to know the landscape of green space scientifically, especially through the analysis and research of synusiologic elements structure of green space on a landscape scale has outstanding advantages. Land synusiologic suitability evaluation is based on synusiologic environmental sensitivity evaluation. Ecological sensitivity refers to the sensitivity of the ecosystem to human activities, which is used to reflect the possibility of synusiologic imbalance and synusiologic environmental problems. Ecological environmental quality evaluation is essentially a pattern recognition problem, that is, the actual monitoring results of the synusiologic environmental quality evaluation index system are compared with the array of corresponding synusiologic environmental quality evaluation standard values, and the synusiologic environmental quality grade corresponding to the standard value array closest to the array of monitoring values is the recognition result of the BP ANN model, that is, the synusiologic environment quality evaluation result of the corresponding area. The synusiologic environmental grade diagram is shown in Figure 2.

The synusiologic environment is a huge, complex, and changeable system, which is not only influenced by various factors of the wetland ecosystem itself but also affected by various factors in the basin. Therefore, when quantitatively evaluating the quality of its synusiologic environment, it is difficult to realize if all the factors involved are listed as evaluation indexes at present, mainly because some factors are difficult to obtain or cannot be quantified. Precipitation temperature and its distribution, vegetation improvement and its community structure, basic topographic features, and spatial pattern, etc. directly affect the stability and natural balance ability of the regional environment and are the basic elements that constitute the synusiologic environment. Appropriate water and heat are the basic conditions for the survival and reproduction of all living things and affect the regional synusiologic environment. Generally speaking, the modules of the network have more biological significance than the whole network. First of all, each OTU in the module can determine its chemical characteristics according to its respective generic or species names. Then, according to the relationship between the characteristics of each OTU, the function of a module can be determined. Landscape pattern analysis is of great significance in green space planning, and the deep cognition of green space on the site is the foundation of scientific green space planning. The analysis of urban synusiologic landscape patterns is the basis of the implementation, management, and planning of green space synusiologic networks.

This paper selects the following indicators to analyze the landscape pattern of green space in the study area:

The number of patches (NP), NP refers to the total number of patches included in a certain patch type or the total number of patches in the whole landscape. The number of patches can reflect both landscape heterogeneity and landscape fragmentation. The calculation principle is

(5) $$\begin{array}{c} NP=N, \end{array}$$

where *N* represents the total number of patches.

Percent of Landscape (PLAND) refers to the percentage of a landscape block type in the total landscape area. The calculation principle is

(6) $$\begin{array}{c} PLAND=\frac{\sum_{j=1}^{n}a_{ij}}{A}\times 100. \end{array}$$

Among them, *i* represents the type of patches, *j* represents the number of patches, *a*_*ij*_ is the area of landscape patches, and *A* is the area of all patches in the landscape. The value range of PLAND is from 0 to 100. When the value of PLAND is equal to 100, there is only one patch type in the landscape. When PLAND approaches 0, this type is particularly rare in the landscape. PLAND is an important index to select the dominant landscape types in the landscape, which can reflect the biodiversity and dominant species in the landscape.

Class area (CA) represents the total area of each landscape type. The calculation principle is

(7) $$\begin{array}{c} CA=\overset{n}{\underset{j=1}{\sum }}a_{ij}\left(\frac{1}{10000}\right). \end{array}$$

Among them, CA is the total area of a certain type of patch in the landscape, *a*_ij_ represents the area of patch *m*^2^, taking *A* as the unit, 555 as the total area of landscape patches, taking hm^2^ as the unit, and *n* as the number of all patches in the landscape.

Patch density (PD), the calculation principle is

(8) $$\begin{array}{c} PD=\frac{N}{A}. \end{array}$$

Among them, *N* is the total number of a certain type of patches in the landscape, and *A* is the total area of a certain type of patches in the landscape. The larger the value, the wider the distribution of this type of patches in the landscape.

The maximum patch index is (*LPI*), which indicates the degree of influence of different types of landscapes on the whole landscape. The calculation principle is shown in the following formula:

(9) $$\begin{array}{c} LPI=\frac{\mathrm{Max}\left(a_{1}\ldots a_{n}\right)}{A}\left(100\right). \end{array}$$

The patch index reflects the impact of human activities on landscape pattern and the calculation principle is

(10) $$\begin{array}{c} LSI=\frac{0.25E}{\sqrt{A}}. \end{array}$$

Among them, *E* is the perimeter of all patches in the landscape and *A* is the area of all patches in the landscape. The more irregular the patch shapes in the landscape, the greater the value of LSI.

The landscape aggregation index is (AI), and the calculation principle is

(11) $$\begin{array}{c} AI=\left\lfloor \overset{m}{\underset{i=1}{\sum }}\left(\frac{g_{ii}}{\max\;-g_{ii}}\right)P_{i}\right\rfloor \times 100. \end{array}$$

Among them, *g*_ii_ is the number of patches of the same type that are connected between *i* types of patches in the landscape, max is the maximum number of patches of the same type that are connected between *i* types of patches, and *P*_*i*_ is the ratio of the number of patches of the type *i* to the total number of landscape patches. The larger the value of AI, it means that this type is about aggregated this landscape.

Eco-sensitivity evaluation is the evaluation of the possibility, scope, and degree of regional synusiologic environmental problems. According to the spatial difference of synusiologic environmental sensitivity, the study area can be divided into an extremely sensitive area, a highly sensitive area, a moderately sensitive area, a slightly sensitive area, and an insensitive area. The stronger the sensitivity of the regional synusiologic environment, the higher the level of land synusiologic suitable use type, and the more restrictions on its improvement and utilization. Training samples are also called expert samples, that is, the “teacher value” of the BP network model, which is usually a matrix composed of several groups of “input-output pairs”. With the improvement of computer techniques, graph theory has been widely used in almost all domains and has achieved unprecedented improvement. Graph theory is a branch of mathematics, taking graphs as the research object. Among them, a graph is a graph composed of a number of given points and lines connecting two points. This graph is usually used to describe a certain relationship between some things. Points represent things, and lines show that corresponding things have this relationship. In the past, the research on the BP ANN model of environmental quality evaluation usually used the national environmental quality standard as the training sample, but for the evaluation of the synusiologic environmental quality of small towns, if the national synusiologic environmental quality standard was used as the training sample, then the synusiologic environmental quality of administrative villages in the small town might be concentrated on one or two levels. As shown in Figures 3–6, this algorithm is superior to the traditional algorithm. With the increase in training times of the improved neural network, the error rate gradually decreases and the prediction accuracy gradually improves.

The algorithm of the BP model learning process consists of two parts: forward propagation and backward propagation. Its basic idea is: in the forward propagation process, the input sample is processed by the hidden layer unit from the input layer and transmitted to the output layer; If the output layer cannot get the expected output vector when using the existing network connection weights and thresholds in the forward propagation, that is, the error function value is large, it will be transferred to the backward propagation. Modern scientific theories and viewpoints such as system mathematics, fuzzy theory, and grey theory hold that numerous and complex influencing factors in the ecosystem have different influences on the synusiologic environment. There are not only primary and secondary points but also some factors that can be ignored. As shown in Tables 1 and 2 and Figures 7 and 8, the network performance of this algorithm is 18% better than that of the traditional algorithm, and the network has reached a certain synusiologic level, which can provide a buffer for the random shock caused by the rigid interaction mode at the customer level.

As a matter of fact, any system containing a certain binary relationship can be simulated by graphs. Whether two points in a graph are connected or not is our main object of investigation. Because this is closely related to what we are concerned about the internal specific relationship between two objects, the straightness of the connecting line in a graph is not the key point of concern. Therefore, the above elements are ignored, and the concept of graphs is produced by mathematical abstraction. Many factors are interrelated and mutually mapped. One factor can be mapped to another factor, and even many factors can be mapped. Therefore, selecting the main, easily accessible, quantitative, and other factors that can be mapped as much as possible as the evaluation index is enough to obtain the evaluation results that are more in line with the actual synusiologic environment quality.

## 5. Conclusions

Around the world, people pay more and more attention to the quality of human settlements. In order to avoid the conflict between land use and nature protection, the construction of a green space synusiologic network, as a new means of green space planning, is helpful to make strategic decisions on existing expenditures (such as land protection and utilization) and future benefits (such as natural resources and quality of life). The system has different characteristics, so its evaluation index system is also different. When applying a neural network to synusiologic environment quality evaluation, for a complex synusiologic environment or ecosystem with many evaluation indexes, the number of hidden nodes or hidden layers of the network can be appropriately increased to improve the learning ability and training effect of the neural network. ANN is a mature modeling means with many advantages. It has specific applications in many aspects, especially in complex large systems like ecosystems. According to the research in this paper, the network performance of this algorithm is 18% better than that of the traditional algorithm, and it is suitable to be widely put into practice.

## Figures and Tables

**Figure 1:** BP neural network structure.

**Figure 2:** Ecological environment level map.

**Figure 3:** Oxygen content in physical process.

**Figure 4:** Oxygen content in synusiologic process.

**Figure 5:** Average deviation rate.

**Figure 6:** RMS error situation.

**Figure 7:** Change of *k* value.

**Figure 8:** Network training results.

**Table 1:** Changes of *K* value.

	0	10	20	30	40	50	60	70	80	90	100
Algorithm	2.7	2.5	1.8	2	0.8	1.4	1.5	2.3	2.1	2.8	3.2
Traditional algorithm	2.2	1.7	2.1	1.5	2.1	2.0	2.5	1.9	1.6	2.1	2.3

**Table 2:** Network training results.

	0	5	10	15	20	25	30	35	40	45	50
Algorithm	3.1	1.4	1.5	2.6	2.5	2.3	1.2	2.2	2.9	3.2	3.5
Traditional algorithm	1.8	2.2	1.2	3.1	2.4	3.3	2.8	1.5	1.9	2.3	1.7

## Data Availability

The figures and tables used to support the findings of this study are included in the article.
